# Spatial Difference of China’s Regional Logistics Development and Construction of Information Network Platform Based on Artificial Intelligence Technology Under the Background of New Economy

**DOI:** 10.3389/fpsyg.2022.871538

**Published:** 2022-07-14

**Authors:** Shajunyi Zhao, Cuijie Xie

**Affiliations:** ^1^School of Management and Economics, North China University of Water Resources and Electric Power, Zhengzhou, China; ^2^Department of Logistics Management, Hebei Jiaotong Vocational and Technical College, Shijiazhuang, China

**Keywords:** new economy, regional logistics, construction of information network platform, artificial intelligence technology, regional economy

## Abstract

Regional logistics is an important part of the regional economy. It plays an important role in optimizing the allocation of regional resources, promoting the upgrading of regional industrial structure, and promoting the sustainable development of regional economy. It is known as the “accelerator” of regional economic growth. Under the background of the expanding regional economic differences in China, this article focuses on the important components of regional economy, researching on regional logistics in different regions. This article focuses on the regional logistics development level, the internal mechanism of regional logistics promoting regional economic growth, the current situation and influencing factors of regional logistics development level differences, and the regional logistics development level differences. The purpose of this article is to study the application of artificial intelligence technology to the spatial difference analysis of China’s regional logistics development and the construction of information network platform under the background of the new economy. In this article, factor analysis is used to construct the index system. The research shows that the intensity of regional logistics connection is significantly enhanced, the regional logistics network is further improved, and a relatively complete multilevel regional logistics network structure is basically formed. In addition, there are great differences in the level of logistics development among regions. The characteristics of the spatial distribution circle in the eastern, central, and western regions are obvious, which is positively related to the economic development, in the Pearl River Delta with the strongest comprehensive competitiveness. The score coefficient of the Yangtze River Delta logistics area is 1.464, and the score coefficient of the northwest logistics weakest area is −0.328. The development of regional logistics can focus on the construction of logistics park, the construction of logistics network system, the progress of regional logistics technology, and the improvement of logistics efficiency. The construction of logistics park is conducive to the integration of regional logistics resources, improves the utilization efficiency of regional logistics resources, forms the economies of scale, and then reduces the transaction cost of the whole region.

## Introduction

The development of a new economy not only causes the continuous establishment of all kinds of new discipline systems but also brings many changes in the theories and methods of the original disciplines, which makes the disciplines continuously expand in the application field and innovate in the application methods (Kuratko et al., 2015; Neumann et al., 2015). Under the background of the new economy, regional integration is gradually strengthened, and information technology is developing rapidly. In the information age, new technologies and new formats are emerging, especially bringing rapid prosperity to e-commerce (cross-border e-commerce) and the express delivery industry. As a new service industry, the modern logistics industry is increasingly valued by all countries in the world (Geng, 2015; Zhu and Lan, 2016). With the deepening of China’s comprehensive reform, the process of new industrialization, informatization, urbanization, and agricultural modernization has been continuously promoted, the pace of industrial restructuring has been accelerated, and the consumption level and personalized demand of residents have been constantly improved (Adil et al., 2021a; Adil et al., 2021b). It is urgent to establish a more perfect, convenient, efficient, safe, and green consumer goods logistics and distribution system to meet the needs of social and economic development. As a basic and strategic industry, logistics industry plays an important supporting role in the development of the national economy, and its industrial status has been significantly improved. With the steady and rapid economic growth and continuous improvement of the development environment, China’s logistics industry has also made great progress (Farouk et al., 2020; Yilin, 2016).

The development level of regional logistics is an important indicator to measure the economic development level of a certain region (Carrillo, 2015; Khalaf and Abdulsahib, 2021). Scientific evaluation of regional logistics development level and analysis of spatial differences and evolution characteristics of regional logistics have important practical significance for improving regional logistics competitiveness, optimizing regional logistics spatial layout, and improving regional economic structure (Hamidi and Jahanshahifard, 2018). At present, the research of foreign scholars on regional logistics mainly focuses on related theoretical research, regional logistics network spatial structure research, and logistics node-related issues. Domestic scholars mainly focus on the evaluation of regional logistics development level, the coordinated development of regional logistics and economy, the planning of regional logistics park, and the evaluation of regional logistics efficiency; the research on logistics spatial organization mainly focuses on the logistics node research of national logistics spatial layout mode, regional logistics spatial structure, and city scale (Bychkov et al., 2016; Ng et al., 2016). On the whole, the scale of the study on modern logistics industry from the perspective of space is mostly a single administrative region of a province or a prefecture-level city, which is lack of exploring the spatial organization of regional logistics across administrative regions from the perspective of logistics linkage (Chu et al., 2018; Zhou et al., 2015). Therefore, exploring the spatial difference and evolution characteristics of China’s regional logistics development in the context of the new economy can enrich the theoretical research of China’s regional logistics spatial organization in the context of the new economy. It can serve the practical needs of China’s regional spatial planning in the context of the new economy (Cai, 2015; Tang, 2016).

The logistics industry is a comprehensive industry integrating transportation, storage, loading and unloading, circulation processing, distribution, and information technology. With the acceleration of economic globalization and integration, logistics has become a new driving force for the rapid development of the national and regional economies. The close relationship between economic development and logistics development is widely concerned by academia. However, most of the current research on the coordination of economy and logistics is focused on the conceptual interpretation and qualitative discussion. Few scholars make quantitative analysis on the coordination of urban economy and logistics. To study this problem, LANS first establishes the evaluation index system of urban logistics and economy to investigate whether there is an interaction between urban logistics and economy (Jiang and Prater, 2015; Lan et al., 2017). Then, entropy weight method and Granger causality test were introduced to evaluate and test the logistics and economic development level of Beijing, Shanghai, Guangzhou, Chongqing, and Tianjin in 2009–2013. From the dimensions of regional economic investment, regional economic capacity and strength finally test the relationship between the three economic subsystems and the three logistics subsystems and further verify the relationship between urban economy and logistics (Cheong and Suthiwartnarueput, 2015). Cheong I systematically summarizes the problems existing in traditional regional logistics and cargo transportation by using the ideas and methods of big data. These problems include data block segmentation in the management system, outdated data collection technology and processing methods, and data resource sharing, which lead to low efficiency and unreasonable layout of regional logistics and freight operation. Cheong I combines the research results of traditional regional logistics and freight development, and studies how to use big data method to establish a modern regional logistics and freight optimization model with the characteristics of volume, speed, change, and value. Cheong’s research purpose is to make the regional logistics and freight layout more reasonable and the management more efficient to provide theoretical and methodological support for promoting regional logistics and freight development (Chen et al., 2016; Wang et al., 2017). Regional logistics demand is the key factor of logistics center location, which changes with the development of regional economy and the change of industrial structure. It is noted that different industries will produce different logistics demand. To study the impact of industry on logistics demand, Chen S models the location of regional logistics hub. Chen S discusses the combination of multicriteria decision-making and integer programming model to solve this problem. The TOPSIS method and mathematical model are used to deal with the qualitative and quantitative factors affecting the location of regional industrial logistics center, and a genetic algorithm is used to solve the problem. Taking the actual data of Sichuan Province as an example, the feasibility of the model and method is verified. The results show that Chengdu, Leshan, and Deyang are selected as comprehensive logistics hub, cross-regional logistics hub, and internal logistics hub, respectively, from 18 candidate cities. The calculation results are consistent with the actual economic and logistics conditions of the study area (Pedrosa et al., 2015; Sun, 2017). To study the internal law of the development of regional logistics network, sun Q analyzes the evolution mechanism, process, and stage of regional logistics network. Second, two evolution models are established by herfindahl-hirschman index and the standard deviation of each logistics node. The time series evolution of regional logistics network is analyzed based on these two models. Through the empirical analysis of the data of Hubei Province, the evolution process and stage of the logistics network in Hubei Province are obtained. The results show that the Wuhan logistics area has the characteristics of hub radiation network, while the Jingyi logistics area and Xiangxi logistics area are still in a low-level equilibrium stage (Sun et al., 2018).

This article uses the factor analysis method, selects nine logistics regions in China as the research object, constructs the index system, calculates the location Gini coefficient and location entropy of the nine logistics regions, and studies the spatial difference and evolution of regional logistics development in China under the new economic background. The research shows that the regional logistics connection strength is significantly enhanced, and the regional logistics network is further improved. The whole multilevel regional logistics network structure is basically formed.

## Proposed Method

### Research Methods

(1) Factor analysis

Factor analysis refers to the study of statistical techniques that extract common factors from groups of variables. Factor analysis allows the identification of hidden representative factors among many variables. Grouping variables of the same essence into a single factor reduces the number of variables and also tests the hypothesis of relationships between variables.

Factor analysis is to group the variables according to the correlation, so that the variables in the same group have a high correlation. That is to say, some variables with overlapping information and complex relationship are reduced to a few uncorrelated comprehensive factors, and most of the information is reflected by a few factors. The calculation formula is:


(1) $$F=\left(\lambda_{1}\,F_{1}+\lambda_{2}\,F_{2}+\cdots +\lambda_{n}\,F_{n}\right)/\sum_{i=1}^{n}\lambda_{i}$$

where *F* is the comprehensive score of the evaluation object; λ_*i*_ is the contribution rate of the characteristic value of each common factor; *F*_*i*_ is the score value of each common factor; $\sum_{i=1}^{n}\lambda_{i}$ is the cumulative contribution rate of the characteristic value.

The main purpose of factor analysis is to describe some of the more basic, but not directly measurable, hidden variables hidden in a set of measured variables. For example, if you want to measure student motivation, active participation in class, homework completion, and reading time outside of class can be used to reflect motivation. The academic performance can be reflected in the mid-term and final grades. In this study, learning enthusiasm and academic performance cannot be directly measured by a measure (e.g., a question), they must be measured by a set of measurement methods, and then, the measurement results can be combined to be more accurately grasped. In other words, these variables cannot be measured directly. What can be directly measured maybe just a representation it reflects or a part of it. Here, representation and part are two different concepts. The representation is directly determined by this implicit variable. Implicit variables are causes, while representations are effects. For example, learning enthusiasm is a major determinant of classroom participation.

There are two types of factor analysis methods. One is exploratory factor analysis and the other is confirmatory factor analysis. Exploratory factor analysis does not presuppose the relationships between factors and measures but lets the data “speak for itself.” Principal component analysis and cofactor analysis are typical methods among them. Confirmatory factor analysis assumes that the relationship between factors and measures is partially known, that is, which measure corresponds to which factor, although we do not yet know the exact coefficients.

Exploratory factor analysis has some limitations. First, it assumes that all factors (after rotation) will affect the measurement term. In actual research, we often assume that since there is no causal relationship between factors, one factor may not affect the measure of another factor. Second, exploratory factor analysis assumes that the residuals of the measurement terms are independent of each other. In fact, the residuals of measurement items can be correlated due to single method bias, subfactors, and so on.

The strength of confirmatory factor analysis is that it allows researchers to explicitly describe the details of a theoretical model. Therefore, what does a researcher want to describe? We have mentioned that because of measurement error, researchers need to use multiple measures. When more than one measure is used, we have the issue of the “quality” of the measure, the validity test. The validity test is to see whether a measurement item has a significant load on its designed factor and no significant load on an irrelevant factor. Of course, we may further test whether there is single method bias in a measurement tool and whether there are “sub-factors” between some measures. These tests require the researcher to explicitly describe the relationship between measures, factors, and residuals. The description of this relationship is also called a measurement model. Quality checking of measurement models is a necessary step before hypothesis testing.

(2) Location Gini coefficient

Location Gini coefficient is an index to describe the distribution degree of an industry in a region. The larger the value is, the more concentrated the industry distribution is. The calculation formula is:


(2) $$G_{i}=\frac{1}{2\,n^{2}\,\mu }\sum_{k=1}^{n}\sum_{j=1}^{n}|S_{i\,j}-S_{i\,k}|\left(j,k=1,2,\ldots ,n\right)$$

where *S*_*ij*_ and *S*_*ik*_ are the shares of regional *j* and regional *k* in industry (*i*or a certain economic activity), μ is the number of regional units, and *n* is the mean value of the shares of each region in the industry (*i* or an economic activity). If only the location Gini coefficient of a certain economic activity is calculated, the subscript *i* in the above formula can be omitted. Generally speaking, the spatial Gini coefficient < 0.20 indicates that the industry is extremely dispersed in space, 0.20–0.30 indicates highly dispersed, 0.30–0.40 indicates relatively dispersed, 0.40–0.50 indicates relatively concentrated, and more than 0.50 indicates highly concentrated.

(3) Location entropy

Location entropy is a quantitative tool for analyzing the efficiency and benefit of an industry. It is used to measure the relative concentration of an industry in a specific area. The calculation formula is as follows:


(3) $$LQ_{i\,j}=\frac{E_{i\,j}/\sum_{i=1}^{n}E_{i\,j}}{\sum_{i=1}^{n}E_{i\,j}/\sum_{i=1}^{n}\sum_{j=1}^{n}E_{i\,j}}\left(i,j=1,2,\ldots ,n\right)$$

where *Eij* is the employment or added value of industrial *j* in *i*; $\sum_{j=1}^{n}E_{i\,j}$ is the total employment or added value of regional *i*; $\sum_{i=1}^{n}E_{i\,j}$ is the employment or added value of industrial *j* in the sample population; $\sum_{i=1}^{n}\sum_{j=1}^{n}E_{i\,j}$ is the total employment or added value of the sample population. Generally, the location entropy is divided into five levels. The high concentration area is > 2.00, the high concentration area is 1.51–2.00, the high concentration area is 1.01–1.50, the low concentration area is 0.51–1.00, and the low concentration area is < 0.50.

### The Connotation of the New Economy

The concept of the new economy first appeared in the United States Business Week. The meaning and characteristics of the new economy can be summarized through three aspects, namely, the knowledge economy is a new socio-economic form; the virtual economy is a new mode of economic activity; and the network economy is a new mode of economic operation.

(1) The characteristics of the new economy in the new socio-economic form of the knowledge economy.

1) Based on knowledge, enterprises from omnipotent production focus on a certain link, process-oriented production, flexible production, the traditional property rights relationship into a contractual cooperation mode of separation of brain industry, and the scope of globalization.
2) The knowledge content in the product is getting higher and higher. Because the marginal cost of knowledge reuse is very low, the higher the technical content in the export product, the greater the actual profit. Products with higher knowledge in international trade account for a larger proportion.
3) Knowledge is the most important factor of production. The degree of concentration of enterprise knowledge represents the core elements and concentration. The more a company grows bigger and stronger, the more it relies on knowledge elements. In the era of industrial economy, capital determines the destiny of enterprises, while in the era of knowledge economy, knowledge and ideas determine the destiny of enterprises.

(2) The characteristics of the new economy in the new economic activity mode of the virtual economy.

1) Complexity. The virtual economic system is a complex system. The non-linear effect between the components in the system is prone to chaos, but the self-organization of the system itself can show certain order and stability.
2) Meta-stability. The virtual economic system is a meta-stable system with a dissipative structure, and each component must exchange material and energy with the external environment to maintain a relative stability. There is also feedback in this process.
3) High risk. The risks of a virtual economy system are high, sometimes unpredictable and unbearable. Due to the certain uncertainty in the virtual operation of enterprises and the limitations of people’s cognitive abilities, many economic activities are one-off, unique, and no precedent can be used for reference.

The development of regional logistics industry is manifested in the transfer of logistics factor resources from low-efficiency departments to high-efficiency departments and the continuous flow of logistics factor resources outside the region into high-efficiency departments in the region. The regional logistics industry development model is a certain industrial development model adopted by a country or region in order to promote the development of the regional logistics industry in the process of developing the regional economy, which embodies the systematic integration of various elements of the logistics industry.

(3) The characteristics of the new economy in the new economic operation mode of the network economy.

1) Information technology is the foundation. Information technology connects businesses, business units, and business functions around the world in a quiet and continuous manner. Make information spread between different business functions, different business organizations, and geographical boundaries like never before and without any trace. The use of information technology plays an important role in helping companies reduce inventory and reduce the cost of core business processes, that is, to produce according to market demand.
2) High transparency and closeness to consumers. The adverse effects of information asymmetry on the operation of the market economy have been largely eliminated. Because the Internet provides a large number of opportunities for producers and consumers in the global economic system to connect directly, consumers have more and more space and freedom to choose their business. Whenever and wherever, they can get what they need by entering the Internet. Various information of products, and through the analysis and comparison of the information provided by different producers, directly select satisfactory personalized needs, the network economy enables enterprises to reduce barriers to market entry, and it is more and more difficult to retain customers. Higher requirements are placed on the level of customer management of the company.
3) High integration. The network economy is an intensive economy. It integrates all aspects of economic activities and all processes through information, so that overall optimization can be achieved. Virtual enterprises have the conditions for their development and growth. As long as the enterprises build a network that links all links of the supply chain, the leading enterprises can transfer the digital drawings of advanced technical specifications design to the technology, assembly, and economy through the network. They are manufactured at the most suitable nodes and assembled directly at the geographically appropriate nodes and delivered directly to the customer. In this way, the resource allocation can be optimized globally, the quality can be improved, the delivery time can be shortened, and a large amount of equipment investment and human resources can be saved, thereby greatly improving the efficiency of management.

The important role of the development of the regional logistics industry on the regional economy is reflected in the following: First, it can reduce costs and improve the efficiency and level of regional economic activities. The continuous refinement of the division of labor objectively helps to improve the level of cooperation, and the development of regional logistics helps to improve the efficiency of resource operation and reduce transaction costs, which is crucial to the efficiency and level of intra-regional economic development and inter-regional economic cooperation. The second influence is to optimize the allocation of resources and promote the adjustment of economic structure.

We are at the turning juncture of the century, and the old economy will eventually be replaced by a new economy that is better suited to the needs of the new era. Therefore, what exactly is the concrete difference between what we call the old and new economies? Obviously, the most fundamental difference between them is that the old economy based on manufacturing was characterized by standardization, scale, patterning, efficiency, and hierarchy, while the new economy was based on information technology. Above all, the pursuit is differentiation, personalization, networking, and speed.

In the stage of regional economic cooperation, that is, the primary stage of regional market development, regional logistics activities are based on the division of labor in primary regions, with the content of adjusting surplus and shortage between adjacent regions and exchanging products. Although there is a prototype based on the overall interests of the region, the influence of administrative regulation still dominates. In the stage of regional economic penetration, that is, the intermediate stage of regional market development, regional logistics activities are based on the deepening regional division of labor and regional specialization, with inter-regional commodity exchange, financial integration, and technical cooperation as the main content, with close characteristics of sexuality, relative stability, and diversity. In the stage of regional economic integration, that is, the advanced stage of regional market development, regional logistics activities are based on the highly developed regional division of labor, with the free flow of all activity elements in the region as the content, forming a regional market structure that is interdependent and highly correlated, and the regional logistics is gradually moving toward integration.

### Basic Concepts of Regional Logistics

(1) The concept of regional logistics

Regional logistics refers to the adaptation of regional environmental characteristics to comprehensively support the overall goal of regional sustainable development, providing regional logistics functions to meet regional economic, political, natural, military, and other development needs, with reasonable spatial structure, service scale, effective organization, and the logistics system of management. The main body of regional logistics is regional cargo transportation. Regional logistics belongs to the category of Zhongguan logistics, which is composed of enterprise logistics, production logistics, and sales logistics belonging to the micro-logistics category. At the same time, the logistics activities system of each region together constitutes a larger regional logistics system, even international logistics. The “region” in regional logistics does not only refer to the division of administrative regions but also refer more to an economic region. Logistics activities are closely linked to production, circulation, and consumption. They are an important part of social and economic activities and a link between social production and social activities. Therefore, the division of logistics areas should consider more the economic development level and characteristics of logistics service areas, and not only the regional boundaries of regional logistics based on geographical boundaries.

(2) Regional logistics center

The “region” of regional logistics mainly refers to an economic region, in which there is often a regional logistics center, which makes the logistics activities of the region closely entangled around it and radiates the region. Therefore, the regional logistics center is often the central city of the entire economic region. The development of a regional logistics is first manifested in the development of its regional logistics center, and the development of the two is closely related. The regional logistics center does not refer to a logistics center, a logistics park, or an integrated distribution center. It is a centralized place for various logistics infrastructures. There are often multiple logistics parks and logistics distribution centers in it. Most logistics operations are handled in the region. The regional logistics center can also be regarded as a logistics node with multiple functions, bringing together the original scattered logistics activities in the entire region, thus realizing the effective use of resources.

(3) Characteristics of regional logistics

1) The “region” in the main diversified regional logistics is an administrative region, an economic region, or a consortium that can be large or small. In this geographical area, there are often a large number of specialized and non-specialized logistics business units. There is competition and cooperation between these units, which makes the logistics market in the region form a complex competitive structure. Moreover, when the “region” in regional logistics is a combination of two or more administrative regions or economic regions, the administrative bodies of regional logistics will also become diversified, and there will be competition and cooperation between them, for example, competition around regional logistics administration rights. This shows that regional logistics has both competition and cooperation between logistics management entities, as well as competition and cooperation between logistics administration entities.
2) The variability of regional boundaries. With the changes in economic resources, industrial structure, information technology, and logistics technology, regional members and regional boundaries in regional logistics will also change accordingly. Changes in the abovementioned regional environment will lead to changes in the size and structure of the region, either expanding (regional economic prosperity) or narrowing (regional economic recession), resulting in changes in the scale and structure of the region. Eventually, the members and regional boundaries of the region change. When the regional economy prospers, the logistics scale of the region will expand accordingly, so that the radiation range of regional logistics, that is, the regional boundaries will also expand accordingly; on the contrary, when the regional economy declines, the logistics scale and regional boundaries of the region will shrink. It has even been integrated into other regions, such as cities with depleted resources. For a “region” of regional logistics with multiple administrative regions or economic regions, changes in the abovementioned logistics environment will change the membership of the region, or the addition of new members, or the withdrawal of the original members. As a result, the boundaries of the region have expanded, shrunk, reorganized, and even disappeared. That is to say, the regional boundaries of regional logistics often change and lack stability.
3) Difficult organization and management, and high cost. Whether it is regional logistics in an administrative region or economic region, or regional logistics in multiple administrative regions or economic regional consortiums, it has a large number of logistics operations’ entities and multiple logistics administrations’ subjects. Therefore, it is very difficult to organize and manage regional logistics, and the cost is also high. This requires regional logistics organizations and managers to explore scientific management methods and management systems, not only to have efficiency concepts, but also to have efficiency concepts. Especially for the logistics administrative managers of large regions composed of multiple administrative regions or economic regions, before adding new members, the organization and management costs of regional logistics and their forms of sharing should be fully considered, and the regions cannot be blindly expanded boundary.

Regional logistics to a large extent refers to regional logistics and local logistics, which mainly have the following basic characteristics, namely, differences in the distribution of spatial resources, differences in the degree of logistics development, relative independence of logistics interests, and integrity of logistics systems.

The difference in the distribution of spatial resources is the economic basis for the formation of regional logistics. Space resources include natural resources and social resources. The distribution of spatial resources in any country or region cannot be completely equal and homogeneous, so in real life, regional logistics shows great differences and diversity. Of course, within a logistics area, there are differences in the distribution of space resources, but they are generally the same; otherwise, it will not become the same logistics area.

The difference in the degree of logistics development is an important criterion for dividing the logistics area. The level of logistics service is always in line with the degree of social and economic development. Therefore, the division of logistics areas is mainly determined according to the degree of economic development, and the degree of economic development mainly examines gross domestic product (GDP), per capita GDP, fiscal revenue, fixed asset investment scale, social consumption level, labor productivity, and other economic indicators.

There is no doubt that regional logistics and local logistics, as subsystems of the regional economic system, are relatively independent economic stakeholders, and each region has its own economic interests. Even economically developed regions have been helped by economically backward regions in natural resources, labor, capital, and other aspects for a long time, and it is obligatory to support and help backward regions after their development.

(4) Classification of regional logistics

Since the concept of “region” in regional logistics is multiple, there are different levels or different scales of regional logistics. This article believes that regional logistics mainly has the following types:

1) International logistics

International logistics refers to the logistics carried out between two or more countries. It is the regional logistics with the highest level, the widest scope, the largest scale, and the most difficult management. The organization and management of international logistics involve many problems, such as the economic system of regional members, international trade policies, business habits, the extension of the hinterland of goods, cultural traditions, the versatility of logistics equipment and tools, the sharing of logistics infrastructure, the standardization of logistics information, and other issues. At the same time, the organization and management of international logistics and its related parties are also very complex, including the central government of the relevant countries, local governments at all levels, logistics demanders, logistics providers, and logistics service intermediaries. Therefore, to solve the abovementioned problems, it is necessary to establish a new international logistics management system to coordinate various relationships, so as to play the role of international logistics in promoting regional economic development.

2) Regional logistics

Regional logistics refers to the logistics of a regional complex composed of several adjacent administrative regions within a country and even national logistics. Regional logistics has large regional boundaries and many regional members, often composed of several provinces. For example, “Northeast Logistics,” “Yangtze River Delta Logistics,” and “Liaohai Sea Area Logistics” all belong to the concept of regional logistics. The reason why large-area logistics can be formed is often because regional members in the region have obvious complementary relationships in terms of industrial structure, industrial division of labor, resource endowment, and geographic location. Therefore, by organizing and developing regional logistics and strengthening logistics cooperation among its regional members, greater social and economic benefits can be obtained. Of course, the formation and development of logistics in some regions are related to history and tradition. For example, the implementation of the revitalization strategy of the old industrial bases in northeast China has further strengthened the links between the three provinces in northeast China and has promoted the formation and development of logistics in northeast China. Due to the large regional boundaries of logistics in the region, there are also many logistics management entities and logistics administrative management entities. Therefore, the organization and management of logistics in large regions are often difficult.

3) Provincial logistics

As the name suggests, provincial logistics refers to logistics within the scope of a province, autonomous region or municipality, such as “Zhejiang Logistics,” “Xinjiang Logistics,” and “Shanghai Logistics.” The area of provincial logistics is a province, autonomous region or municipality, but in a province, it is highly probable that small- and medium-sized regional logistics consists of several municipal, county, district, and other administrative regions within the province. Compared with regional logistics, the organization and management of provincial logistics are relatively difficult, because even if there are a number of low-level regional logistics in the province, because they are administratively affiliated to a province, the policy is relatively uniform. These low-level regional logistics are also relatively easy to coordinate.

4) City logistics

Urban logistics refers to logistics activities that serve urban social and economic development and focuses on regional logistics research. The main feature of urban logistics is the unified management and management of all logistics activities in the city. Moreover, compared with regional logistics, such as international logistics and regional logistics, the regional scope of urban logistics is relatively small. Therefore, urban logistics has a very strong controllability. The long-term development of a city is based on the establishment and development of a city logistics system. After the city has formed a certain scale, the economic activities of the entire city are based on logistics. A city’s long-term development plan not only requires direct planning of logistics infrastructure and logistics projects, such as the construction of roads, tunnels, bridges, and warehouses, but also requires the use of logistics as a constraint to plan the entire city, such as factories, residential areas, stations, and airports. Reasonable urban logistics can efficiently supply all kinds of materials needed for production and living in the entire city. At present, logistics has become a key part of the planning and construction of all large cities in the world.

5) Rural logistics

Rural logistics is a concept corresponding to urban logistics. It refers to the logistics that serves the rural areas and the rural residents. There was also a suburban logistics concept between urban logistics and rural logistics. However, from the perspective of many domestic and international logistics practices, suburban logistics should be attributed to urban logistics. This is because with the rapid development of urbanization and industrialization in cities, urban logistics outlets, especially urban logistics centers, have the trend of shifting to the suburbs. Therefore, in this sense, suburban logistics itself is an important part of urban logistics.

## Experiments

### Data Sources and Research Methods

The data used in this article were collected from the 2012 to 2018 China Statistical Yearbook, the China Economic and Social Development Statistics Database, the 2012 to 2018 China Transportation Yearbook, and the 2012 to 2018 provincial and municipal statistical yearbooks.

### Research Objects

The purpose of this article is to study the spatial differences and evolution of regional logistics development in China under the background of new economy, and to study the nine major logistics regions in China. The layout of the nine major logistics regions in the country is as follows: (1) North China logistics area centered on Beijing and Tianjin; (2) northeast area logistics centered on Shenyang and Dalian; (3) Shandong Peninsula logistics area centered on Qingdao; (4) the Yangtze River Delta Logistics Regional Center centered on Shanghai, Nanjing, and Ningbo; (5) the southeast coastal logistics area centered on Xiamen; (6) the Pearl River Delta logistics area centered on Guangzhou and Shenzhen; (7) in Wuhan, Zhengzhou is the central logistics area; (8) the northwest logistics area centered on Xi’an, Lanzhou, and Urumqi; and (9) the southwest logistics area centered on Chongqing, Chengdu, and Nanning.

### Index System Construction

According to the data availability, comparability and comprehensive index selection principles, and drawing on relevant research results, this article constructs regional logistics from five aspects, namely, economic development level, logistics demand status, logistics industry scale, information level, and infrastructure construction. Comprehensive development-level indicator system is shown in Table 1.

**TABLE 1:** Regional logistics industry comprehensive development-level index system.

Target layer	Criterion layer	Index layer
Comprehensive logistics development level	Economic development level	GDP (10^8^yuan), Per capita GDP (10^8^yuan)
	Logistics demand	Gross industrial output value (10^8^yuan), Total value of farm output (10^8^yuan), Total retail sales of social consumer goods (10^8^yuan), Total freight volume (10^4^t)
	Logistics industry scale	Added value of logistics-related industries (10^8^yuan), Number of logistics employees (10^4^people)
	Level of information	Total postal services (10^8^yuan), Number of Internet users (10^4^household), Number of mobile phone end users (10^4^household)
	Infrastructure construction	Inland waterway mileage (10^4^km), Highway mileage (10^4^km), Length of railroad lines in service (10^4^km), Air carrier capacity, Total investment in fixed assets in logistics (10^8^yuan)

## Discussion

### Evaluation of the Development Level of Comprehensive Indicators

Factor analysis of the 2017 indicator data in Table 1 is carried out by using formula (1), and three principal components are extracted. According to the main component score and variance contribution rate, the comprehensive scores of the logistics development level of the nine major logistics regions are obtained. The results are shown in Figure 1.

**FIGURE 1:** The comprehensive score of the nine major logistics areas.

As can be seen from Figure 1, the nine logistics areas are classified as follows: The first level is the first category (comprehensive score > 0), including North China Logistics area, Northeast Logistics area, Shandong Peninsula Logistics area, Yangtze River Delta Logistics area, Pearl River Delta logistics area, and Southwest Logistics area. The second level is the second category [comprehensive score (−0.2, 0)], including the central logistics area. The third level is the third category [comprehensive score (−0.2, −0.4)], including the southeast logistics area, the central logistics area, and the northwest logistics area. It can be seen that the regional differences in the level of regional logistics development are obvious. The Pearl River Delta logistics area with the most comprehensive competitiveness has a scoring coefficient of 1.464, and the weakest northwest logistics area has a scoring coefficient of −0.328.

### Analysis and Evaluation of the Level of Competitiveness

The level of competitiveness of the nine major logistics regional logistics was calculated in 2015 and 2017, that is, the average of the comprehensive factor scores of the provinces included in each logistics area as the level of logistics competitiveness of the region was used, and the levels of logistics competitiveness of the nine regional regions were ranked, as shown in Figure 2.

**FIGURE 2:** Analysis of the level of competitiveness of the nine major logistics regions.

Generally speaking, the higher the comprehensive factor score of each logistics area, the stronger the logistics competitiveness of the region. The score greater than 0 indicates that the level of logistics competitiveness of the region is above the average level of the nine logistics regions. Less than 0 indicates that the level of logistics competitiveness of the region is below the average level of the nine major logistics areas. It can be seen from Figure 2 that the level of competitiveness development is gradually increasing in the Pearl River Delta area, the Yangtze River Delta area, the North China region, and the southeast coastal region, while the competitiveness is gradually decreasing in the Shandong Peninsula region, the northeast region, the central region, the southwest region, and the northwest region.

### Logistics Industry Location Gini Coefficient

The distribution of regional logistics is relatively concentrated, and the trend of agglomeration has evolved from enhanced to weakened. Using the number of employment personnel in the logistics industry of various provinces and cities to enter the formula (2) to calculate the Gini coefficient of the logistics industry in the nine major logistics areas from 2012 to 2018, the results are shown in Figure 3.

**FIGURE 3:** Gini coefficient of logistics business in the 2012–2018 logistics area.

It can be seen from Figure 3 that the Gini coefficient of the logistics industry in China’s nine major logistics regions increased from 2012 to 2018, and fluctuated after reaching a peak of 0.4589 in 2015. In 2012, the Gini coefficient of the location was between 0.3 and 0.4, and the regional logistics spatial distribution was in a relatively dispersed state. In other years, the Gini coefficient of the location was between 0.4 and 0.5, which was in a relatively concentrated state. In general, the distribution of logistics space in the nine major logistics regions is in a relatively concentrated state and has undergone an evolution process from decentralization to concentration. The concentration trend shows a strong first and then weak.

### Logistics Industry Location Entropy

The logistics industry location entropy is calculated by using the number of logistics employment personnel and the total number of employed persons in the nine major logistics areas (3). The results are shown in Figure 4.

**FIGURE 4:** Location entropy of the logistics industry in the nine major logistics regions.

The coexistence of spatial agglomeration effect and dispersion effect makes the difference of regional logistics agglomeration degree between provinces expand continuously. It can be seen from the figure that the location entropy of the Pearl River Delta fluctuates from 1.05 to 1.37, which belongs to a higher industry agglomeration area; the location entropy of the Yangtze River Delta fluctuates from 1.15 to 1.36, which belongs to a higher industry agglomeration area; the location entropy of the Shandong Peninsula fluctuates from 1.05 to 1.16, which belongs to a higher industry agglomeration area; the location entropy of the North China region fluctuates from 0.98 to 1.17, which changes from a lower industry agglomeration area to a row. The location entropy of the northeast region fluctuates from 0.95 to 1.05, which changes from a lower industry cluster to a higher industry cluster; the location entropy of the southeast coastal region fluctuates from 0.98 to 1.13, which changes from a lower industry cluster to a higher industry cluster; the location entropy of the central region fluctuates from 0.89 to 1.03, which only exceeds 1.0 in one year, which belongs to a lower industry cluster; the regional entropy of Northeast China fluctuates between 0.95 and 1.05, which belongs to the lower industry cluster area; the regional location entropy fluctuates between 0.65 and 82, which belongs to the lower industry cluster area.

## Conclusion

With the rapid development of the world economy, the global logistics industry is facing severe challenges. While the industry competition is more intense, the division of labor is also more detailed. At the same time, with the further innovation of electronic information technology, the analysis of modern logistics mode has also set off a new wave. Modern logistics develops in the direction of informatization, modernization, and intelligence. Combined with the international logistics form, the progress of modern logistics should always focus on serving consumers, forms a unified and perfect logistics service operation mode, and promotes its continuous improvement and progress, so as to further promotes the realization of the economic benefits and social development interests of logistics enterprises.

Under the background of new economy, this article makes a preliminary study on the application of artificial intelligence technology in the spatial difference analysis of China’s regional logistics development and the construction of information network platform. Through the calculation of the single index and comprehensive index of the logistics development level of nine regions, it is found that there are great regional differences in the logistics development level of China under the background of new economy. The spatial distribution characteristics of the three eastern regions are significantly different in the central and western regions, which is positively related to economic development. Among them, the Pearl River Delta logistics region with the strongest comprehensive competitiveness has the weakest score coefficient, which is 1.464. The score coefficient of the northwest logistics area is −0.328; at the same time, modern logistics is also facing huge development opportunities and challenges. As an important part of regional economy, regional logistics plays an important role in optimizing the allocation of regional resources, promoting the upgrading of regional industrial structure, and promoting the sustainable development of regional economy.

This article made a comprehensive evaluation on the logistics competitiveness of the nine logistics regions in 2012 and 2018 by factor analysis, and analyzed the changes of their logistics competitiveness. The results show that the Pearl River Delta and Yangtze River Delta still maintain a strong level of logistics competitiveness. In recent years, the logistics industry in the central and southwest regions has developed rapidly, especially in the central region, omic levels in different regions also show different characteristics.

## Data Availability Statement

The original contributions presented in this study are included in the article/supplementary material, further inquiries can be directed to the corresponding author.

## Author Contributions

SZ: editing data curation and supervision. CX: writing – original draft preparation. Both authors contributed to the article and approved the submitted version.

## Conflict of Interest

The authors declare that the research was conducted in the absence of any commercial or financial relationships that could be construed as a potential conflict of interest.

## Publisher’s Note

All claims expressed in this article are solely those of the authors and do not necessarily represent those of their affiliated organizations, or those of the publisher, the editors and the reviewers. Any product that may be evaluated in this article, or claim that may be made by its manufacturer, is not guaranteed or endorsed by the publisher.

## References

[B1] AdilM.KhanM. K.JamjoomM.FaroukA. (2021a). *MHADBOR: AI-Enabled Administrative Distance Based Opportunistic Load Balancing Scheme for an Agriculture Internet of Things Network.* Piscataway: IEEE Micro.

[B2] AdilM.SongH.AliJ.JanM. A.AttiqueM.AbbasS. (2021b). EnhancedAODV: A Robust Three Phase Priority-based Traffic Load Balancing Scheme for Internet of Things. *IEEE Inter. Things J.* [Epub online ahead of print] 10.1109/JIOT.2021.3072984

[B3] BychkovI. V.KazakovA. L.LempertA. A.BukharovD. S. (2016). An intelligent management system for the development of a regional transport logistics infrastructure. *Automat. Remote Control* 77 332–343.

[B4] CaiW. (2015). Development of Western Logistics Finance Based on Village Banks:A Case Study of Baise City in Guangxi. *Asian Agric. Res.* 7 40–43.

[B5] CarrilloF. J. (2015). Knowledge-based development as a new economic culture. *J. Open Innovat. Technol. Market Complex.* 1:15.

[B6] ChenS.ChenD.GanM. (2016). The Regional Logistics Hubs Location Problem Based on the Technique for Order Preference by Similarity to an Ideal Solution and Genetic Algorithm: A Case of Sichuan. *J. Computat. Theor. Nanosci.* 13 6065–6075.

[B7] CheongI.SuthiwartnarueputK. (2015). ASEAN’s initiatives for regional economic integration and the implications for maritime logistics reforms. *Int. J. Logist. Manag.* 26 479–493.

[B8] ChuX.SuX. X.CaiF.ChenJ. (2018). An efficient auction mechanism for regional logistics synchronization. *J. Intell. Manufact.* 30 2715–2731.

[B9] FaroukA.AlahmadiA.GhoseS.MashatanA. (2020). Blockchain platform for industrial healthcare: vision and future opportunities. *Comput. Commun.* 154 223–235.

[B10] GengW. (2015). The viscous analysis on inter-district transfer of textile industry from the perspective of New Economic Geography in China. *Geogr. Res.* 34 259–269.

[B11] HamidiH.JahanshahifardM. (2018). The Role of the Internet of Things in the Improvement and Expansion of Business. *J. Organ. End User Comput.* 30 24–44.

[B12] JiangB.PraterE. (2015). Distribution and logistics development in China. *Int. J. Phys. Distr. Logist. Manag.* 32 783–798.

[B13] KhalafO. I.AbdulsahibG. M. (2021). Optimized dynamic storage of data (ODSD) in IoT based on blockchain for wireless sensor networks. *Peer Peer Netw. Appl.* 14 2858–2873.

[B14] KuratkoD. F.HornsbyJ. S.HaytonJ. (2015). Corporate entrepreneurship: the innovative challenge for a new global economic reality. *Small Bus. Econ.* 45 245–253.

[B15] LanS.ChenY.HuangG. Q. (2017). Data analysis for metropolitan economic and logistics development. *Adv. Eng. Inform.* 32 66–76.

[B16] NeumannJ. E.EmanuelK.RavelaS.LudwigL.KirshenP.BosmaK. (2015). Joint effects of storm surge and sea-level rise on US Coasts: new economic estimates of impacts, adaptation, and benefits of mitigation policy. *Clim. Change* 129 337–349.

[B17] NgA. K. Y.YangZ.CahoonS.LeeP. T. W. (2016). Introduction: port, Maritime Logistics, and Regional Development. *Growth Change* 47 346–348.

[B18] PedrosaA. D. M.BlazevicV.JasmandC. (2015). Logistics innovation development: a micro-level perspective. *Int. J. Phys. Distr. Logist. Manag.* 45 313–332.

[B19] SunB.LiH.ZhaoQ. (2018). Logistics agglomeration and logistics productivity in the USA. *Ann. Region. Sci.* 61 273–293.

[B20] SunQ. (2017). Empirical research on coordination evaluation and sustainable development mechanism of regional logistics and new-type urbanization: a panel data analysis from 2000 to 2015 for Liaoning Province in China. *Environ. Sci. Pollut. Res.* 24 14163–14175. 10.1007/s11356-017-8980-y 28421518

[B21] TangL. (2016). Problems in Development of Rural E- commerce and Logistics and Recommendations. *Asian Agric. Res.* 8 41–47.

[B22] WangP.ZhangX.JieH. E.HanB.YangH. China Railway Corporation (2017). Research on Hierarchical and Dynamic Location Optimization for Railway Automobile Logistics Bases under Business Mode of “Forward Stocking”. *J. CHIN. Railway Soc.* 39 1–9.

[B23] YilinW. (2016). Chinese Energy Enterprises’ Transformation and Development under China’s New Economic Normal. *CHIN. Oil Gas* 23 3–4.

[B24] ZhouL.GuZ.ZhaoG.LuoJ. (2015). Calculation and Evaluation of Carbon Dioxide Emissions of Regional Logistics Ecosystem: A Study in China. *Nat. Environ. Pollut. Technol.* 88 1227–1236.

[B25] ZhuS.LanT. (2016). New economic geographies of manufacturing in China. *Geogr. Compass* 10 470–481.

